The article "Multiscale Layout and Planning of Smart Gardens in the Environment of Agricultural Internet of Things" was published in 2022. Journal: Comput Intell Neurosci.

# Multiscale Layout and Planning of Smart Gardens in the Environment of Agricultural Internet of Things

**DOI:** 10.1155/2022/4746629

**Published:** 2022-04-25

**Authors:** Xiuting Geng, Ou Chun

**Affiliations:** School of Life and Food Engineering, Fuyang Normal University, Fuyang, Anhui 236037, China

## Abstract

This paper studies the general architecture and key technologies of the Agricultural Internet of Things and summarizes the latest progress of the Internet of Things system model. On this basis, a general system architecture model suitable for the Agricultural Internet of Things is initially established, and the key technologies of the Agricultural Internet of Things are expounded to provide a reference for the in-depth application and development of the Agricultural Internet of Things. Aiming at the problem that the energy consumption of each node in the network is uneven in the process of monitoring agricultural production environment by wireless sensor network, which leads to the failure of some nodes in the network too fast, an event-driven wireless routing algorithm for agricultural production environment monitoring is proposed. By reducing the number of pieces of control information sent in the cluster, the algorithm selects the next hop forwarding node from candidate nodes according to the forwarding cost function to shorten the data transmission distance, reduce energy consumption, and improve the life cycle of the entire network. The experimental results show that the algorithm in this paper effectively avoids the waste of node energy consumption caused by the active transmission mode and at the same time better balances the overall energy consumption of the network and prolongs the life cycle of the network. The platform satisfies the needs of a local garden bureau to integrate comprehensive landscaping business information and display comprehensive landscaping information in a comprehensive, timely, and dynamic manner. At the same time, it has made useful explorations in the development and integration of landscaping business data interfaces and GIS data interfaces. All system functions of the smart garden information management platform project are reasonably designed and completely correct and basically meet the software function requirements specified in the requirements specification. Some functions were found not realized during the test. After rectification, various systems have been improved. All system interfaces of the smart garden information management platform project have reasonable layout, simple operation, and good ease of use. The smart garden information management platform project meets the business logic requirements and fulfills the requirements of the information construction of the Garden and Greening Administration. All systems of the smart garden information management platform project are simple to install and easy to operate and meet the user's requirements after installation. The system has a strict permission setting function. People with different permissions can only see the content of the fields that they have permission to access, which effectively ensures the security of the data.

## 1. Introduction

In recent years, the government has vigorously advocated “Internet+,” combining traditional industries with Internet thinking to promote the development of the real economy, bringing opportunities and challenges to the garden industry [1]. However, there are information asymmetry in the original industrial chain, low utilization rate of resources, low standardization, primitive transaction process, prominent contradiction between supply and demand, difficult transformation of scientific research achievements, weak capital gathering force, lack of professional and technical personnel, and weak scientific popularization in the industry [2]. As far as Guangzhou is concerned, the industry authorities are still in the stage of policy guidance and exploration of “Internet+ gardens”; botanical gardens focus on collecting plant resources and have little research on application. Talent cultivation is the main focus; scientific research institutes focus more on their own advantageous research fields or some “short, flat, and fast” greening projects, lack of motivation for research on public welfare and common issues, and the transformation efficiency of scientific research results. It is also relatively low; even if the company has made some explorations on the individual common problems of the industry, it is also out of consideration for its own interests [3]. Although the industry information website has released some cutting-edge information and supply and demand information, it lacks credibility. The main bodies of the industry have only carried out partial explorations for their own functional areas or business scope and have not been able to effectively integrate the advantageous resources of all parties to form a joint force for industry development [4].

Good landscaping management is the cornerstone and guarantee of urban landscaping work. With an efficient and scientific landscaping management system, people's pressure can be relieved, which is beneficial to human health and improves people's sense of happiness [5]. It is a powerful guarantee for the construction of ecological civilization. “Smart garden, dream garden” has become an inevitable trend in the development of modern gardens, and the construction of garden informatization is gradually changing the survival and operation mode of the garden industry [6]. It will further make the landscaping management more information-based and intelligent and reduce the cost of garden construction, and the work efficiency will also be greatly improved. Scholars use computer technology, 3S technology, and network technology to establish a comprehensive landscaping digital information system that is suitable for popularization and convenient for public participation and attention and closely integrates digital information technology with landscaping management to serve landscaping management and improve management [7]. Efficiency, optimization of management effects, and realization of automated, intelligent, and scientific management are urgent and important issues [8]. With the development of green urbanization construction and “smart gardens,” digital information technology is gradually applied in urban landscaping construction. Studying the application of digital information system in landscaping management will provide a certain scientific basis for landscaping management [9].

This paper constructs the architecture model of the Agricultural Internet of Things, that is, through comprehensive perception and, data transmission to heterogeneous data aggregation, using the expert decision-making model to provide feedback control, and constructing a unified public service platform for agricultural producers, consumers, and governments. Specifically, the technical contributions of this paper can be summarized as follows:

First, because wireless sensor network has the characteristics of low cost, low power consumption, high reliability, self-organization, and so on, it has been widely used in agricultural production environment monitoring systems. However, it also has inherent limitations of wireless transmission media, such as low transmission bandwidth. The transmission process is prone to errors, channel conflicts, and so on, these nodes are deployed in the wild, even in places that humans cannot reach, which makes the sensor nodes only rely on limited batteries for power supply, and some nodes close to the base station are easy to transmit due to heavy transmission tasks. It leads to the failure of the node, which leads to the failure of the wireless monitoring in the area it is responsible for. The cluster head node always communicates directly with the sink point, and this paper proposes an event-driven wireless monitoring method for agricultural production environment. By reducing the number of pieces of control information sent in the cluster, the algorithm selects the next hop forwarding node from the candidate nodes according to the forwarding cost function to shorten the data transmission distance, reduce energy consumption, and improve the life cycle of the entire network. The simulation experiment is carried out by OMNET++ simulation software, and the results show that the algorithm in this paper can better solve the problem of unbalanced network energy consumption and prolong the life cycle of the network.

Second, the smart garden operation and maintenance support system is mainly a background management system used by platform administrators. It will realize the management of various online services of the platform (data directory service, data service, functional service, etc.), the management and scheduling of user rights, and the status monitoring and quality evaluation of services, service access statistics, and other functions. The platform can provide secure and stable support for various client application access. The landscaping comprehensive resource management system is mainly used by data administrators. It follows the special data standards for landscaping and develops and realizes the functions of checking, warehousing, updating, and outputting comprehensive landscaping resource data. In the design and development of the entire smart garden information management platform, while participating in the overall design, the author divides labor to design and implement the smart garden comprehensive information portal part of the platform, that is, to realize the monitoring of garden attractions, monitoring of world cultural heritage, landscaping project information monitoring, video monitoring, and other information interfaces, as well as map query, statistical analysis, and other functions.

## 2. Related Work

The hierarchical structure of the Internet of Things consists of three layers, which are sensors, transmission networks, and application services. Developed countries in foreign countries have applied these three layers to the agricultural field, from crops to seedlings, to production, and finally to harvesting and storage [10]. The process utilizes the sensor technology to the fullest extent. Foreign universities, research institutes, and well-known enterprises have made outstanding contributions to the research on the Agricultural Internet of Things. Farmers from left to Asia were already using long-range video systems and GPS to monitor the agricultural field environment [11]. In terms of wireless networks, many universities in the United States have carried out a lot of research work [12]. Among them, the University of California, Los Angeles, has established a forestry resource and environmental monitoring network, which improves the real-time monitoring and effective utilization of resources and provides huge technical support for the overall management of forestry [13]. In terms of agricultural ecological monitoring, the United States, France, Japan, and other countries have been able to combine advanced sensing technology, using information fusion technology and Internet technology and other high-tech means to establish agricultural ecological monitoring networks. A variety of Internet of Things application service standards have been established, and in some fields, it has occupied a leading position in the industry [14].

At present, the research and application of digital information systems are developing at an astonishing speed, and such high-speed development marks the substantial progress of information technology [15]. Digital information systems have been widely concerned and applied by governments at all levels and the industry abroad. Especially in countries and regions such as Europe, North America, Japan, and Australia, digital information systems have basically formed a market [16]. Now the digital information system data companies and software companies on the market are springing up one after another, which proves that the digital information system is relatively mature in many aspects, and the application is also very standardized [17].

Singapore is a typical representative of the government's self-built model. Singapore's e-government system is completely funded by the state, without the participation of any social forces, and a series of highly targeted measures have been formulated during the construction process to ensure the health of the platform. The Japanese government, on the other hand, has solved the problem of informatization development by adopting a unified bidding method from the central to local governments, which not only effectively avoids duplication of construction and waste of resources but also improves the efficiency of the use of resources such as funds and information [18]. Japan has a lot of experience in the construction of e-government. It has established an information processing center to serve the surrounding areas of radiation and linkage and has fixed staff to solve relevant technical problems in a timely manner, responsible for data security and daily maintenance of the platform.

Relevant scholars integrate various high-quality resources scattered in the government, scientific research institutions, colleges and universities, enterprises, intermediary service agencies, and the public on the basis of respecting the development law of the garden industry itself [19]. Relevant scholars take innovation, coconstruction, and sharing construction mechanism as the core and aim at integrating and opening up industry resources, improving efficiency, and providing support to build a basic, open, professional, and nonprofit industry aggregate and improve the level of industry public services and services [20].

Relevant scholars pointed out that, due to its own public welfare and administrative functions, the garden industry determines that the public service platform of the garden industry does not have the conditions for market-oriented operation, which requires the construction subject to include the government, scientific research institutions, enterprises, intermediaries, and other forces and resources [21–23]. The platform cannot adopt a single market-oriented model but adopts a four-in-one model of “government-led, scientific research institute-led, enterprise coconstruction, and alliance collaboration,” which is more suitable for the current stage of development. The identity and nature of the participating subjects will have a series of direct impacts on the policy orientation, platform construction mode, and operation mode because the subject is an important implementer who comprehensively integrates the latest scientific research achievements and technical services in the industry and successfully transforms and promotes it. In the process of implementation, through information technology, network technology, database technology, and so on, the garden industry participants in the province and even the whole country will be more widely linked, and a strong subject cluster will have better resistance to risks. At the same time, the breadth and depth of the integration of industry resources will determine the success or failure of platform construction [24–26]. Therefore, it is necessary to not only comprehensively and effectively integrate relevant information and resources but also integrate the concepts of industry participants.

## 3. Methods

### 3.1. Architecture of Agricultural Internet of Things

We synthesize the goals and requirements of the application of IoT technology in the agricultural field and build a general architecture model suitable for the agricultural IoT. The model is divided into perception layer, transmission layer, and application layer (data aggregation, analysis and decision-making, and application services). The overall architecture of the agricultural IoT platform is shown in Figure 1.

The perception layer is like the “skin” and “facial features” of the Internet of Things, which are mainly responsible for recognizing objects and collecting information. Common sensing devices include environmental information sensors, RFID tags and readers, meteorological data monitors, cameras, and GPS devices. The main task of this layer is to convert physical quantities such as agricultural production in the real world into digital information that can be analyzed and processed in the virtual world in real time through various means.

In the production process of agricultural products, with the help of environmental and soil monitoring sensors and visual video data, data support is provided for the safety supervision of agricultural products.

In the Agricultural Internet of Things, the network layer is required to transmit the data sensed by the perception layer quickly, reliably, and safely. It solves the problem of data transmission obtained by the perception layer. At the same time, the network layer will undertake more data volume and face higher quality requirements than the existing network. The network constructed in the agricultural field cannot yet meet the needs of IoT applications. It is necessary to fully integrate and expand the existing network and adopt new technologies to achieve extensive and efficient transmission functions. The main task of this layer is to aggregate the collected agricultural data information through various network technologies and methods so as to realize the integration of information for further analysis and processing. The network application technologies involved in the information aggregation layer include wired network and wireless network.

WSN is an important means of sensing things and transmitting data in the Agricultural Internet of Things, just like the important “tentacles” and “nerves” of the Internet of Things. Using WSN's features such as self-organizing network, low power consumption, scalability, low cost, and low complexity, the data of smart sensors, environmental monitoring instruments, and other types of equipment are incorporated into the wireless network, and various data can be quickly transmitted back to the central server. The device transmission module supports the connection of various analog and digital smart sensors; the built-in lithium polymer battery and the self-developed sleep/wake system can support the device to work for a long time and can be easily charged. The module can self-organize the network, and the whole network can be expanded so that the equipment can be used in a large scale.

The application layer is mainly based on the characteristics and needs of various agricultural industries, using Internet technology and means to develop application solutions suitable for the agricultural industry. Combining the technical advantages of the Internet of Things with agricultural production and operation, information management, and organization scheduling, various Agricultural Internet of Things solutions are formed to meet common and individual application needs.

### 3.2. Event-Driven Energy-Efficient Clustering Routing Protocol

The entire sensor network needs to be initialized and configured after the first deployment. In order to obtain the distance between each node and the BS node, the BS node broadcasts the S_ADV message using the flooding mechanism, and each node estimates the distance between itself and the BS node according to the received signal strength indicator (RSSI). In this protocol, the nodes can obtain the distance from other nodes by exchanging the request to establish a cluster message (REQ_CLUSTER) or the request to forward the node message (REQ_RELAY).

In order to save energy, after the network initialization is completed, all nodes enter the sleep state. When an event is detected, the dormant nodes around the event are activated and obtain specific information of the monitored data.

If the sensed information exceeds a preset threshold, the activated nodes run the cluster establishment and cluster head election algorithms. All activated nodes broadcast REQ_CLUSTER data packets (including node ID, remaining energy, and descriptive information of the perceived data in the event) to other activated nodes to request the establishment of a clustering network.

Assuming that *n* nodes are activated, if all nodes send broadcast messages, the number of broadcast messages sent is *n∗*(*n* − 1) times. This protocol randomly selects an activated node elector to send a broadcast message and waits for all other nodes to return the response information RES_CLUSTER; then, the total number of sent and received messages is 2*∗*(*n* − 1). After the elector node receives all the response information, it compares and sorts the remaining energy of all nodes. The node with the most remaining energy is elected as the cluster head (CH) and forwards the IDs of all cluster member nodes to CH, and the node with the next elector energy is the next node. If the elector's energy is more than the remaining energy of other nodes after the round, the probability of the elector becoming the cluster head node in the next round will further increase, reducing the transmission of more response messages.

After the cluster head node is elected, the cluster head allocates the TDMA scheduling plan according to the number of cluster members in this event and broadcasts TDMA_MSG data packets to the member nodes in the cluster to ensure that each node transmits sensing data to the cluster head node in an orderly manner.

We assume that the BS node is far away from each sensor node, so the cluster head node must transmit the fused data to the BS node through the forwarding node (also called the relay node). The fused data are sent to the BS node. Using the TDMA schedule, each node transmits sensing data to the cluster head node in its allocated time slot. In order to save energy, each node is in a dormant state before the time slot allocated for each node arrives and is only in an active state and transmits data in its allocated time slot.

Compared with data transmission, data processing consumes much less energy, so intracluster data processing is very important to reduce data redundancy and save transmission energy. After the cluster head node collects the data of all members in the cluster, it executes the corresponding data fusion algorithm, thereby reducing the amount of data sent to the BS node.

The cluster head node that wants to send data first checks whether the BS is within its communication range. If it is, it directly sends the data to the BS. If it is not within its communication range, the cluster head broadcasts a request to forward (REQ_RELAY) to the nodes within its communication range. REQ_RELAY packet contains node ID, remaining energy, and distance information from BS. The node that receives REQ_RELAY will decide whether to return the response forwarding (RESPON_RELAY) packet according to the distance between itself and the BS and the distance between the requesting node and the BS in REQ_RELAY, and only the candidate node closer to the BS needs to make the response. The response packet contains information such as node ID, end-to-end average delay, remaining energy, and distance from the sink node. After the cluster head node receives the response packet from the neighbor node, it selects the next hop forwarding node from the candidate nodes according to the forwarding cost function.

(1) $$\begin{array}{c} F_{RN}\left(j\right)=\frac{\text{Delay}\left(CH,j\right)}{E_{res}\left(j\right)}•\frac{d\left(j,BS\right)}{d\left(CH,j\right)}. \end{array}$$

The node with the largest value among all candidate nodes will be selected as the forwarding node. In the next hop, the forwarding node acts as the cluster head to find the next forwarding node, and this process is repeated until the next hop is the BS node. Finally, an optimal transmission path from the cluster head node to the BS node is established.  Figure 2 depicts the flowchart of the data transfer phase.

### 3.3. Genetic Algorithm Planning of Garden Site Selection Problem

Chromosomes are composed of the most basic genetic material “genes” according to a certain arrangement, and several consecutive genes constitute a gene fragment, which contains several characteristics of a species. It is the chromosomes contained in the individuals in the population that carry out “crossover,” “mutation,” and “selection” aimed at adaptability in the process of evolution so that the “excellent” gene fragments carried by the excellent individuals in the population are more numerous. It has been strengthened, so that better individuals can be combined, and the population also shows the characteristics of continuous evolution from low level to high level.

For individuals, the rules followed in evolution are fairly simple: species evolve under the action of natural selection (through crossover, mutation, or other forms), and the more adaptable the individuals are, the easier it is to survive and reproduce. The “genetic material” is copied to the next generation. It is this simple individual rule that enables continuous evolution of excellent individuals in the group.

The number of individuals in a group is called the size of the group, also known as the population size. The degree of adaptation of each individual to the environment is called fitness, which indicates the degree to which the chromosomes possessed by the individual can solve the problem. In algorithm evolution, individuals with high adaptability can produce more excellent offspring, forming positive feedback on population evolution.

Assuming that the number of *H* patterns in the population at time *t* is expressed as *m*(*H*, *t*), the average fitness of all individuals with *H* patterns is *µ*(*H*, *t*), and the expected number of *H* patterns at time *t* + 1 is *E*(*m*(*H*, *t* + 1)); according to the roulette selection algorithm, the expectation of chromosome *x* entering the next generation is *f(x*)*/f* ′(*t*).

Among them, *f*(*x*) represents the fitness of chromosome *x*, and *f* ′(*t*) is the average fitness of the entire chromosome group at time *t*; only considering the selection operation, then

(2) $$\begin{array}{c} E\left[m\left(H,t-1\right)\right]=m\left(H,t\right)•\frac{u\left(H,t\right)}{f^{\prime }\left(t\right)}. \end{array}$$

Considering the influence of crossover, when the probability of crossover is *P*_*c*_, then the probability *S*_*c*_(*H*) that mode *H* can survive to the next generation is

(3) $$\begin{array}{c} S_{c}\left(H\right)=1-\frac{d\left(H\right)}{n+1}•P_{c}. \end{array}$$

Among them, *d*(*H*) is the defined length of the pattern *H*, and *n* is the length of the search space string. It can be seen that the shorter the pattern is, the easier it is to survive. Similarly, when the mutation probability is *P*_*m*_, use *S*_*m*_(*H*) to represent the probability of *H* survival under the action of mutation; then, we have

(4) $$\begin{array}{c} S_{m}\left(H\right)={\left(P_{c}-P_{m}\right)}^{O\left(H\right)}, \end{array}$$

where *O*(*H*) is the rank of *H*, that is, the number of characters determined in the pattern string. It can be seen that under the action of mutation, the mode with lower rank is more likely to survive.

In order to facilitate the calculation, the research space is transformed into a discrete grid space. Define *P* as a point set in a 2-dimensional plane space as a research space. Generally, this space includes a garden demand point set *R*, a fixed garden facility point set *S*′, and a planning garden facility candidate point set *S*″.

(5) $$\begin{array}{c} P=\left(\begin{array}{cccc} p_{0} & p_{1} & \cdots & p_{m-1} \end{array}\right)P=S^{\prime }\cap R\cap S^{'\prime }. \end{array}$$

Suppose there are *x* garden demand points in the space, and define the garden demand point set:

(6) $$\begin{array}{c} R=\left(\begin{array}{cccc} r_{0} & r_{1} & \cdots & r_{x-1} \end{array}\right)R=S^{\prime \prime }\cap P. \end{array}$$

Suppose there are *k* existing garden facilities, and define the fixed garden point set as

(7) $$\begin{array}{c} S^{\prime }=\left(\begin{array}{cccc} s_{0}^{\prime } & s_{1}^{\prime } & \cdots & s_{k-1}^{\prime } \end{array}\right)S^{\prime }=P_{c}\cap P. \end{array}$$

There are *n* candidate points, and the candidate garden point set is defined as

(8) $$\begin{array}{c} S^{\prime \prime }=\left(\begin{array}{cccc} s_{0}^{\prime \prime } & s_{1}^{\prime \prime } & \cdots & s_{n-1}^{\prime \prime } \end{array}\right)S^{\prime \prime }=P_{m}\cap P. \end{array}$$

The garden demand point set *R* consists of *y* entities of the garden responsibility area that can be divided, and *E* is the entity set. It forms a partition on *R* that satisfies

(9) $$\begin{array}{c} \left\{\begin{array}{c} R=\prod_{i=0}^{y-1}e_{i}\\ e_{i}\cup e_{j}\notin \emptyset -1<i,\;j<y-1 \end{array}\right). \end{array}$$

## 4. Results and Analysis

### 4.1. Test Environment and Configuration

The test environment and operating environment configuration of the smart garden information management platform include the configuration of hardware environment, network environment, and software environment. The hardware environment is mainly to establish and debug the server, client, peripherals, and other hardware environments for system operation; the network environment plays the role of connecting the server and the client to ensure the normal operation of the system; the software environment refers to the server and the client.

The server segment is configured with one database server and two web servers; the client is configured with several PCs and a set of large-screen systems. The network links with other business application systems are mainly located in the same set of government affairs network, and the multiple servers of other businesses can be connected to each other, but the direct communication with other business application systems is mainly maintained in the form of service interfaces. The configuration of the platform hardware is shown in Table 1.

The test method is mainly functional test, which takes the functional module defined in the functional requirement specification as the unit. The focus of functional testing is whether the main functions of each system can be used normally. The system test focuses on checking whether the page link is correct, checking whether the function of the button is correct, checking the string length, checking the character type, checking the integrity of the information brought out, repeating the information, checking the required items, checking the shortcut keys, and browser compatibility. In addition, it also includes interface testing, regression testing, and installation testing.

### 4.2. Algorithm Simulation Experiment

When there are a small number of sensing nodes in the sensor network, the physical measurement experimental method can be used to evaluate the performance of the sensing network. However, with the continuous growth of the wireless sensor network scale, especially the large-scale wireless sensor network containing a large number of nodes, the physical experimental method becomes unsustainable. With the emergence and development of computer network simulation software, network simulation through computer has become the main means to test the performance of wireless sensor network routing protocol algorithms.

Although Network Simulator-2 (NS-2) includes a large number of tools for routing algorithm and TCP protocol simulation, it is mainly used for OSI model simulation, and NS-2's simulation of packet level is close to runtime. Therefore, it is not well suited for large-scale network simulation.

Because NS involves a lot of content, it is necessary to master a lot of related knowledge and tools to conduct simulation tests. Objective Modular Network Testbed in C++ (OMNeT++) as a discrete event network system simulator supports Windows, Linux, Mac OS X, and other systems. Based on the Eclipse platform, it provides a complete integrated development environment with a complete visual graphical interface, which is convenient for users to use. Therefore, this paper uses the OMNeT++ network simulator to simulate the improved EDEEC wireless sensor network protocol algorithm.

In order to verify the feasibility and effectiveness of the EDEEC routing algorithm, the EDEEC, LEACH, and ARPEES protocols are simulated in the OMNET++ simulation software. Each node is evenly distributed in a 500 × 500 square area, the base station is set at (250, 500), and the energy is not limited. Set the initialization energy of all nodes to 1.5 J (Joules), and other simulation parameters are set as shown in Table 2.

The network life cycle of the three algorithms is shown in Figure 3. The ordinate is the number of remaining surviving nodes in the network, and the abscissa is the number of rounds performed by the network. As can be seen from the figure, the network life cycle of the algorithm in this paper is the largest. Compared with the ARPEES algorithm and the LEACH protocol algorithm, the algorithm in this paper effectively prolongs the lifetime of the entire network.

It can be seen from the comparison between Figures 4 and 5 that when the algorithm in this paper uses data fusion, the number of surviving nodes at the same time of rounds is more than that of LEACH and ARPEES. It can be seen that, at the same time, there are more surviving nodes after the survival node fusion algorithm in this paper, and the packet loss rate of the data becomes smaller, so the algorithm in this paper has a certain reference value.

### 4.3. Test Content and Result Analysis

The test is carried out in strict accordance with the project plan and test plan, and the test of the test objects specified in the test plan is completed. The test strategy specified in the test plan is reflected in the test execution. In the process of test execution, each function point of the two systems of the smart garden information management platform is completely tested according to the test plan. The test content includes the following four aspects:

1. Functional test: The testers performed all the use case points listed in the test case, and the actual results of each use case were recorded in detail.
2. User interface testing: User interface testing and functional testing are done concurrently. In the process of interface testing, features such as ease of use, standardization, rationality, aesthetics, and coordination are taken into account, and the requirements of users are met.
3. Regression testing: The testers executed all the regression test cases and made detailed records of the actual results of each use case. In the regression test, it is confirmed that the developers have fixed all the bugs submitted by the testers, and no exceptions were found.
4. Installation test: The installer has been tested under Windows 10 operating system.

Requirements coverage refers to the ratio of the tested requirements/functions to all requirements/functions in the requirements specification, usually the 90% target. The demand coverage is shown in Figure 6.

The smart garden information management platform integrates multiple business application systems of landscaping in a certain area, including electronic ticket management system, dynamic supervision information system of scenic spots in a certain area, dynamic monitoring information system of world cultural heritage, dynamic information system of landscaping enterprises, and landscape tourism network. At the same time, it realizes the connection with the basic geographic information sharing service platform in a certain region, and the integrated sharing calls the basic geographic information. At present, the interface calls between the various systems are smooth and smooth, and the dynamic data of various landscaping topics can be obtained quickly, comprehensively, and timely through a platform, which makes it easy for the leaders and managers of the landscaping bureau to have a comprehensive grasp of the city's landscaping dynamics. The statistical results by defect source and severity are shown in Figure 7. The statistical results by defect repair rate are shown in Figure 8. In the first round of testing, the defect discovery rate reached 94%, and after multiple regression tests, the defect discovery rate reached 100%. The use case quality and defect density all meet the requirements.

A smart garden information management platform has been installed and deployed in the command and monitoring center of the Garden Bureau, which can be implemented on the big screen: quick browsing of the city's maps and query and browsing of the data and distribution of landscaping thematic maps. On the big screen, you can view the real-time surveillance video of the specified camera in the form of a list and select camera points on the video surveillance distribution map. You can view the dynamic monitoring information of classical gardens (world cultural heritage) in a certain area and so on. At present, the system is running in good condition, ensuring 24-hour monitoring.

For example, the staff of the security department use the smart garden information management platform on a daily basis to comprehensively monitor the real-time status of key gardens and park scenic spots in a certain area and protect the gardens and park scenic spots from man-made damage. The system can monitor the passenger flow and publish the number of people in the park in real time. When a certain value is reached, the system can issue a warning and early warning, and through the video camera, the passenger flow in and around the scenic spot can be viewed in real time.

At the same time, for emergencies or major activities, the system can quickly call out the preset emergency command and dispatch plan to avoid congestion or more serious situations. The system is in good condition in the security department and other garden bureau departments.

## 5. Conclusion

In the era of rapid development of information technology, there can be no modernization without informatization. Agricultural informatization has become one of the important symbols of agricultural modernization, and informatization is the commanding height of agricultural modernization. Whether it can win the initiative in the application of the Agricultural Internet of Things not only is related to the improvement of agricultural comprehensive production capacity and international competitiveness but also will become one of the important productivity factors affecting the development of agricultural and rural economy. As the key technology of Agricultural Internet of Things monitoring, wireless sensor network has incomparable advantages over traditional monitoring networks. However, due to the limited energy of sensing nodes, some nodes close to the base station are prone to node failure due to heavy transmission tasks. Aiming at the problem that the traditional LEACH routing algorithm assumes that the sensor node continuously sends data to the cluster head node and the cluster head node always communicates directly with the rendezvous point, an event-driven energy-efficient clustering routing protocol algorithm is proposed. Simulation experiments are carried out to evaluate the performance of the algorithm proposed in this paper. The experimental results show that the proposed algorithm can better solve the problem of unbalanced network energy consumption and prolong the life cycle of the network.

The smart garden information management platform integrates GIS, the Internet of Things, and so on in technology and realizes the sharing and integration of multisource, multiscale geographic data, and structured data through application system interfaces and GIS-shared service interfaces. It has realized flexible and diverse comprehensive information inquiry of landscaping; in terms of business, it has integrated many businesses such as garden tickets, emergency security, key projects, heritage monitoring, and video surveillance in landscaping management, forming a comprehensive, timely, and comprehensive landscaping business information. The smart garden information management platform initially realizes the aggregation and collaboration of thematic data sharing services of various departments within a regional garden bureau, at the same time realizes information sharing with other commissions, offices, and bureaus, and finally builds a set of scientific and standardized urban geographic information sharing services. The carrier, cross-departmental comprehensive information, and comprehensive three-dimensional landscaping informatization service system meets the needs of quick query and acquisition of comprehensive landscaping information and real-time dynamic information through large screens, computers, and so on, so as to effectively improve the city's gardens. The information dynamic update ability, heterogeneous resource aggregation ability, ubiquitous real-time service ability, and comprehensive information sharing ability of greening topic information resources meet the increasing urgent needs of urban planning, construction, management, and the public for comprehensive information on greening topic. It provides strong support for the construction of a “smart region” that is livable, suitable for industry, and suitable for travel.

## Figures and Tables

**Figure 1:** Organizational structure of the Agricultural Internet of Things.

**Figure 2:** Flowchart of the data transfer phase.

**Figure 3:** Life cycle comparison of routing algorithms.

**Figure 4:** When there is no data fusion, the node survival rate changes with the number of rounds.

**Figure 5:** When data is merged, the node survival rate changes with the number of rounds.

**Figure 6:** Requirements coverage.

**Figure 7:** Defect source statistics.

**Figure 8:** Defect repair rate statistics.

**Table 1:** Platform hardware configuration.

Serial number	Hardware name	Model	Configure	Use
1	Database server	IBM x3850M2	Standard 32 GB DDR2 memory	Also doubles as a map server
2	PC	ASUS	CPU: 2.70GHz RAM: 8 GB	Test client
3	Database server	IBM x3850M2	Standard 32 GB DDR2 memory	Implement mutual backup and proper load balancing
4	Web server	IBM x3850M2	Standard 32 GB DDR2 memory	Deployment platform server-side system software

**Table 2:** Network simulation parameter settings.

Parameter	Value
Control packet size	30 bytes
Perceived range	85 m
Node initial energy	1.5 J
Free channel model transmission energy consumption	9 pJ/bit/m^2^
Number of data frames sent per round	12
Number of simulated transfers	20
Packet size	240 bytes
Transmission range	90 m
Total number of nodes	120
Node death threshold	0.05 J

## Data Availability

The data used to support the findings of this study are available from the corresponding author upon request.
